The article "The Effect of a Theory-Based Educational Intervention on Reducing Aggressive Behavior among Male Students: A Randomized Controlled Trial Study" was published in 2022. Journal: Biomed Res Int.

# The Effect of a Theory-Based Educational Intervention on Reducing Aggressive Behavior among Male Students: A Randomized Controlled Trial Study

**DOI:** 10.1155/2022/6308929

**Published:** 2022-08-23

**Authors:** Mohammad Hossein Kaveh, Ehtesham Ghaysari, Leila Ghahremani, Elahe Zare, Hale Ghaem

**Affiliations:** ^1^Research Center for Health Sciences, Institute of Health, Department of Health Promotion, School of Health, Shiraz University of Medical Sciences, Shiraz, Iran; ^2^Department of Health Promotion, Faculty of Health, Shiraz University of Medical Sciences, Shiraz, Iran; ^3^Research Center for Health Sciences, Institute of Health, Department of Epidemiology, School of Health, Shiraz University of Medical Sciences, Shiraz, Iran

## Abstract

**Introduction:**

One of the most challenging issues in public health is preventing aggression and violent behavior, generally in the adolescent population. Intervention studies in this field, especially in Iran, were few. Moreover, their findings are controversial. Therefore, this study was conducted to investigate the effect of educational intervention based on the theory of planned behavior (TPB) on reducing aggression among male students.

**Method:**

This study used a randomized controlled trial design. The sample comprised 98 middle school students aged between 13 and 16 years (14.28 ± 0.7). Educational intervention for the experimental group consisted of five sessions of 45-60 minutes. Data were collected using two self-administered questionnaires to measure aggression and constructs of TPB. Data were analyzed using paired *t*-test, independent *t*-test, and chi-square test at a significance level of 0.05.

**Results:**

After the intervention, the experimental group showed a significant increase in all TPB constructs except the subjective norms, compared to the control group (*p* < 0.001). After two months of intervention, the mean score of the aggression behaviors in students in the experimental group showed a remarkable improvement in the experimental group, while the control group showed no significant difference.

**Conclusion:**

The findings of this study showed that the theory-based educational intervention was effective on the improvement of aggressive behavior. To achieve a significant change in perceived mental norms, more training sessions are recommended, and emphasis is placed on educating parents, peers, and school staff.

## 1. Introduction

Aggression is the most important risk factor in psychopathology and is a sign of disorders among adolescents and is one of the most common and uncomfortable behaviors among deviant behaviors in humans [1, 2]. In psychology, the term aggression refers to overt verbal or physical behaviors that can lead to physical and psychological harm to oneself, others, or objects in the environment which are seen as predictors of more serious youth violent behaviors [3, 4]. This behavior is manifested in various forms such as shouting or pushing and even more serious actions such as hitting, kicking, or punching to more severe actions such as stabbing, shooting, or killing [5] .Aggressive behavior and violence have serious negative outcomes including anger, anxiety, guilt, shame, delinquency behaviors, social isolation, violence, and academic failure in the future [6–8].

Both Western and Eastern countries are faced with this serious mental health problem [9], because studies have shown that there is a significant relationship between aggression and ideation of suicide and depression. It also causes drug abuse and delinquency and violation of the rights of others [10, 11]. Recent studies in several countries have shown that the prevalence of such behaviors among adolescents has increased [12, 13]. A review study in India found that 17.7% to 66.5% were involved in physical aggression and it was also high (56.8%) for verbal aggression [14]. Another study done by Bucur et al. [15] found that 35.87% of teenagers have taken part in a physical fight during the previous 12 months.

There are gender differences in various kinds of aggression [16]. Evidence found physical aggression to be more among boys and verbal aggression was more in girls [17–19]. The results of one study on gender differences in aggression using electroencephalography (EEG) and electrocardiography (ECG) analysis showed that physical and reactive/overt aggression was stronger in men. In addition, aggressive videos revealed prominent gender-related patterns in *γ*-signals [20]. As well as, Fahlgren et al. reported that aggression was significantly related to trait anger only for male [21].

It is noteworthy that aggressive behavior tends to peak during middle school years [22], because during this period of life, there is significant brain growth in the areas that make up processes related to reactive aggression, such as threat assessment, self-control, and decision-making [23].

Aggression is influenced by a series of individual, academic, family, and social variables in adolescence [19]. Among the risk factors at the individual level that are effective in creating aggressive behaviors are low self-esteem and low life satisfaction. At the school level, factors such as negative attitudes towards school and school staff and negative social relationships with classmates can also be mentioned. At the family level, factors such as lack of emotional cohesion among family members and negative economic and social conditions were effective in the occurrence of aggressive behavior [20]. Even, parental support can have a positive effect, especially in relation to adolescent cognitive development and behavior in the school environment [4]. Almost half of all disciplinary referrals in schools are due to arguing with a teacher or principal or failing to comply with an instruction given by a teacher and aggressive behaviors [21]. The study done by Poling et al. showed the relationship between parental psychological control and adolescent aggression [22]. In addition, exposure to community violence has been reported as one of the risk factors affecting aggression in adolescents [24].

Research depicted that peers have a dramatic influence on aggressive behaviors during adolescence [4, 25]. Peer pressure becomes more difficult to resist in adolescence, because the views of peers are often more important than those of parents. When adolescents form relationships with people who present aggressive behaviors, they were likely to engage in these behaviors themselves. Therefore, if a significant individual engages in aggressive behavior, the adolescents may behave in the same way. Also, if adolescents spend time with deviant peers who use drugs, do not go to school regularly, and are physically aggressive, they were more likely to take part in aggressive behaviors [26]. Hence, a person's attitude towards aggressive behavior is influenced by the attitude and behaviors of proaggression among their peers [27].

Another factor affecting aggression is social norm because the person's decision in high-risk situations is so relevant to the extent that individuals believe that others in their immediate environment would approve or support such behaviors [28]. The study by Finigan-Carr et al. showed that parental support plays a positive role in the lives of adolescents because it can help mitigate the effects of negative economic and social conditions on adolescent aggressive behavior [4]. Evidence has shown that students who receive a sense of respect and support from friends, peers, and teachers in the school environment express a positive attitude towards school and teachers and have not usually exhibit behavioral problems such as aggression [12].

Prevention is important in early adolescence because during this time dating and norms of behavioral are formed [29]. School can be an unrivaled opportunity to implement and evaluate the effectiveness of juvenile aggression prevention education programs [30]. Many prevention strategies include surveillance (e.g., metal detectors and guards) and deterrence (e.g., disciplinary rules and zero tolerance policies). And there are psychosocial programs, with many schools reporting that they use one or more of these prevention strategies to deal with behavioral problems [31]. Also, the results have shown that many schools use mental health strategies, social services, and prevention services for students and their families. However, there is little indication that these school-promoted programs are widely adopted or, once adopted, are faithfully implemented [32]. Evidence has shown that RTC studies have been effective in reducing aggressive behavior [29, 33, 34]. Waschbusch et al. pointed in meta-analytic study of school-based interventions that a theory of change be used for the intervention in order to decide on the proximal goals of the intervention as well as on the methods of achieving better goals and also recommended that it is better to use experimental interventions so that we can better adapt the values or culture of a school [35].

Due to the adverse and multiple consequences of aggression in adolescents, especially in terms of psychosocial health in adulthood for instance, behaviors such as sexual assault, driving and shooting, road rage and hitting, and more serious forms of violence [36], it is necessary to identify appropriate intervention [37]. Effective education and public awareness-raising are fundamental strategies for preventing aggression and violence [38]. Individual empowerment and the development of personal skills, as emphasized in the Ottawa Charter on Health Promotion, are fundamental steps in aggression prevention programs [39]. Various factors, including identifying and targeting behavior determinants through appropriate planning and based on scientific theory and evidence, affect the effectiveness of educational programs [40]. Health education is a helpful strategy that bridges the gap between information and health behaviors. There may be many obstacles to changing behavior, in which theories and educational models are responsible for identifying these factors and adapting them to existing cultural and social factors [41]. Theories of behavior change have played a constructive role in identifying determinants of aggressive behavior and are a useful guide to designing educational interventions [42].

According to the available evidence, individual and interpersonal determinants play a role in the occurrence of aggressive behavior [43–45]. In the present study, theory of planned behavior (TPB) was selected as a framework for planning the intervention and evaluating its impact. TPB is one of the models of behavior change that is well known and predicts the occurrence of a particular behavior [42]. Several studies have shown the ability of TPB to predict aggressive behavior [4, 46, 47]. This theory was used to identify behavioral determinants or to design educational interventions in various areas of health, including low-consumption snacks, watching TV, and using the brush and dental floss, and physical activity has been used [48, 49]. According to TPB, intention and behavior are under the influence of attitudes and subjective norms and perceived behavioral control. It also describes perceived behavioral control based on a person's belief in an individual ability to perform the behavior and how easy or difficult it is to perform that behavior [50]. The construct of TPB helps us better examine interpersonal factors, especially primary groups such as family, peers, and friends [4] and individual factors such as a person's attitude and belief. So it seems that this theory can be used for the design and evaluation of educational intervention. The goals of educational intervention based on TPB were to (1) minimize aggressive behavior and prevent the onset of aggressive behaviors among students, (2) increase students' knowledge about issues related to aggression, (3) increase students' knowledge about the impact of peers and family on aggressive behaviors, (4) train and practice essential skills, (5) create positive attitudes in participants to control anger and manage emotions, and (6) increase students' perceived ability or self-confidence to perform learned skills in controlling and preventing aggression.

While several theoretical explanations for applying the extended TPB model to aggression have been proposed [47, 51, 52], only a limited amount of empirical evidence that supports the application of the TPB to the study of aggression behaviors has been reported thus far. This study was aimed at investigating the effect of theory-based educational intervention on reducing aggression behavior among male students in Bushehr city.

## 2. Materials and Methods

### 2.1. Study Design and Participants

The present study was a randomized controlled trial design that was conducted on male students aged 13 to 16 years in 2016 in Bushehr city, Iran. The sample size was determined by using the following formula [53], based on similar previous study [54], in which the mean score and standard deviation of the study objectives in the intervention and control groups were, respectively, 24.56 ± 3.39 and 20.93 ± 5.24. Also, considering the error of the first type 5%, the test power was 80% with 95% confidence, and taking into account the loss of samples, the sample size was set as *n* = 98 where each of the intervention and control groups had *n* = 49.

(1) $$\begin{array}{c} n=\frac{{\left(Z_{1-\left(\alpha /2\right)}+Z_{1-\beta }\right)}^{2}\left(\delta_{1}^{2}+\delta_{2}^{2}\right)}{{\left(\mu_{1}-\mu_{2}\right)}^{2}}. \end{array}$$

Participants were selected by selected multistage cluster sampling. For this purpose, in the first phase, we randomly selected four schools from list of public schools (*n* = eighteen) in Bushehr city and then randomly assigned two schools to the intervention and two schools to the control group. Finally, randomly one class selected in each school and invited students' participation in the study. In order to prevent data contamination between the intervention and control groups, random allocation was done at the cluster (i.e., school) level. Inclusion criteria were being an eighth-grade male student, regular attendance at school, have informed consent, no history of taking sedatives, and did not attend other educational and therapeutic classes at the same time. Exclusion criteria were students who have not to want to participate in the study and students who did not attend more than two sessions.  Figure 1 presents the CONSORT diagram of the study.

The participants have voluntarily entered the study in order to comply with ethical principles, the study was approved by the Research Council of Shiraz University of Medical Sciences, and related permission was obtained from Bushehr County Department of Education. All participants were informed about the quality of the project implementation, the confidentiality of information, and the purpose of the project, and their written informed consent was obtained. As well as, the informed consent was signed by their parents. Participants were also assured that their information would remain confidential.

### 2.2. Research Tools

Data were collected using two self-administered questionnaires before and two months after the completion of educational intervention in the studied groups. The first part of the first questionnaire included demographic information (student's age and parents' levels of education and occupations). The second part used aggression questionnaire developed by Buss and Perry [55]. This questionnaire evaluates four types of aggressive behaviors (physical, verbal, anger, and hostility) and a self-report tool that contains 29 phrases in a completely different 5-degree spectrum (5), is somewhat similar to me (4), not it looks like me, not like me (3), it is not like me (2), and it is not like me at all (1), and the whole score was obtained with the total score of the subscales. Content validity and reliability of the Persian version of this questionnaire were confirmed by Samani [56]. In the present study, alpha was 0.78 which indicates the good internal reliability of the questionnaire.

The second one was a researcher-made questionnaire that was designed using valid scientific sources [47, 57] to the determinants of aggression behavior using TPB. It was consisted of 57 items of a five-point Likert scale from totally agree to totally disagree (score from 1 to 5) designed and used. In this questionnaire, the attitude was measured with 20 items (for example, in general, when it comes to anger, it is a mistake to deal with others physically), higher scores indicate a negative attitude towards aggression and, subjective norms using 6 items (for example, if someone beats me, my family expects me to beat them) were measured. The perceived behavioral control construct consists of 26 items (for example, it is easy for me to stop the verbal argument), and the ultimately behavioral intention to aggression was measured and used, consisting of 5 items (for instance, I want to learn how to manage my self-anger). The knowledge measuring tool was 30 questions. Out of the thirty questions, six of them were multichoice types (scoring from 0 to 1). The correct answer was given a score of one, and the wrong answer was given a score of zero. Twenty-four of the other questions were asked (yes, no, and I do not know). The score was from 0 to 1, which had the correct answer for score 1 and the false answer had zero scores (for example, listening greatly to control anger). Its content validity was confirmed by a group of health promotion and psychology specialists (*n* = 10). Also, CVR = 0.73 and CVI = 0.86 confirm the validity of this tool [58]. Its reliability was determined by conducting a pilot study and calculating Cronbach's alpha coefficient. Cronbach's alpha coefficient was calculated as 0.681 in knowledge construct, 0.753 in attitude, 0.723 in perceived behavioral control, 0.692 in subjective norms, and 0.781 in behavioral intention.

### 2.3. Intervention

The educational intervention for the experimental group included five sessions, and each session took about one hour. The sessions were delivered over a period of 1 month with one session each week by giving presentations, group discussions, asking and answering questions, presenting educational films and images, and power points. The educational programs were performed by MSc of health education and promotion. How to complete the questionnaire was explained to the students, and the questionnaires were filled out before and two months after the educational intervention by experimental and control groups. Since the number of questions in the questionnaires was large, and filling them in one session may affect the answers; it was decided that the students would complete the questionnaires in two consecutive days. First, the aggression questionnaire and demographic information were completed, and the next day, the TPB-based questionnaire was completed. The details of the training sessions are shown in Table 1. The student of control group received no educational program. They were only asked for filling out questionnaires. At the end of study, one educational session about aggression management skill was held for control group, too.

### 2.4. Statistical Analysis

Data were analyzed using SPSS16 software at significance level of 0.05. First, the normality of data was tested using the Shapiro-Wilk test (*p* ≥ 0.5). Demographic variables were compared between two groups with the chi-square test. Constructs of TPB were compared between two groups with an independent *t*-test. Also, the mean scores of the two groups on aggression behaviors and TPB constructs were compared via paired samples *t*-test before and after the intervention.

## 3. Results

The participants in this study were 98 students. The mean (SD) age of the participants was 14.49 ± 0.77 years in the intervention group and 14.06 ± 0.56 years in the control group. Chi-square test showed that there was no statistically significant difference between the two groups of test and control in terms of fathers' education, mother's education, father's job, and mother's job (Table 2).

The results indicated that based on independent *t*-test, before the intervention, there were no significant differences between the mean scores of TPB constructs in experimental and control groups, except for the perceived behavioral control. However, there were significant differences between the two groups, except for the subjective norm construct two months after the intervention (*p* < 0.001). Paired sample *t*-test showed that mean scores of knowledge, attitude, perceived behavioral control, and behavioral intention increased in the experimental group (*p* < 0.001). In the control group, the mean scores of these constructs did not change significantly (Table 3).

According to Table 3, Cohen's *d* as effect size coefficient indicates the high effectiveness of the intervention in this study, which had a higher effect coefficient belonging to knowledge (Cohen's *d* = 1.97).

In within-group analysis, there were no significant differences in control groups after the intervention in the mean scores of verbal aggression, physical aggression, hostility, and anger; however, in the experimental group after the intervention, the mean score of verbal aggression, physical aggression, hostility, and anger showed significant enhancement than the control group (*p* < 0.001). This result could indicate they have more reducing or controlling aggressive behavior skills in the experimental group (Table 4).

According to Table 4, Cohen's *d* as effect size coefficient indicates the high effectiveness of the intervention in this study, which had a higher effect coefficient belonging to score of anger among students (Cohen's *d* = 0.56).

## 4. Discussion and Conclusion

This study was conducted with the aim of reducing aggression and controlling aggression behaviors while improving attitudes, subjective norms, and perceived behavioral control among male students in Bushehr.

Due to the limited interventional studies in the field of aggressive behaviors based on TPB, it is referred to intervention studies based on this theory but in other research topics.

This study showed that the intervention and control groups did not differ meaningfully from the point of view of demographic variables. The absence of differences between the studied groups from the point of view of demographic variables showed that the stages of the study, including sampling, were done with high and appropriate accuracy and the confounding effect and demographic variables were controlled. Therefore, the attribution of changes observed in the intervention group is powerful.

The results of the study showed that in the experimental group, the mean score of knowledge related to aggression after the intervention was significant. However, there was no significant difference in the control group. This finding is consistent in line with several studies on young adults and adolescents that show that educational intervention programs have increased the individual's knowledge in the experimental group [59, 60], also, corroborated the findings of Khaleghi et al. [61].

There was no significant difference in attitudes between the experimental group and the control group before the intervention. Although, after the intervention, no significant increase in attitude was shown in the adolescents of the experimental group. But, the average scores of this group indicate a negative attitude towards aggression. This finding may be because the educational intervention had an effect on modifying the correct attitude towards aggression in the participants of the intervention group. In the control group, the average scores indicate their positive attitude towards aggression. This result is in line with those reported by Sainsbury et al. [62] and Bai et al. [63].

As the findings of the present study indicated, the mean subjective norm score of the experimental group had no significant difference after the educational intervention, compared to that of the control group. These results agreed with some studies such as Zhao et al. [64] and Jalambadani et al. [65], while in the results of the study, Shalmaii et al. had a significant increase in the subjective norms of the group after intervention [66]. Subjective norms are more influenced by the judgment of others, including parents, siblings, friends, and teachers. To achieve a significant change in perceived mental norms, more training sessions are recommended, and emphasis is placed on educating parents, peers, and school staff.

Also, the results of the present study showed that the mean behavioral intention score related to aggression in the experimental group after the intervention was significantly different. However, in the control group, the mean score of behavioral intention in relation to aggression before and after the intervention was not significant. The results of other studies were consistent with the results of this study [59, 67, 68].

The mean score on perceived behavioral control in the present study showed that before the intervention, students had a low ability to control aggression, while after the intervention, the mean score on perceived behavioral control increased significantly. However, there was no significant difference in the control group. This is consistent with the results of Karimy et al. [69] and Didarloo et al. [70]. The individual intends to perform a behavior when he realizes that the behavior is under his or her control. Sense of control will make them strive to succeed in what they want [67].

Verbal aggression is reactive and overactive to other cases of aggression that were studied in this study. This aggression is defined as a defensive response to perceived stimuli of intimidation or stimulus-inducing enmity [71]. The results of this study showed that verbal aggression was significantly different in the experimental group after the intervention, while there was no significant difference in the control group. Studies have shown that those who believe that aggression is an appropriate response were more aggressive than those who considered aggression to be inadequate or unacceptable in a social situation [4]. In the present study, physical aggression was also studied, and the results showed that the mean scores of physical aggression in the experimental group after the intervention were significantly different. However, there was no significant difference in the control group. The results of this study are consistent with the results of studies by Fares et al., Hirshfeld et al., and Özabacı [72–74]. In this study, the parameters of anger and hostility were also studied. Results showed that there was a significant difference after the intervention. In a study by Vakili et al., the results showed that the level of verbal violence and anger among Spanish students was high [75]. It seems that education in schools can be an important means to reduce anger among students.

In current study, Cohen's *d* as effect size coefficient indicates the high effectiveness of the intervention in this study (*d* = 0.56). But, the results of a meta-analysis showed that school interventions reduce aggression with small effect sizes (*d* = 0.21) [76]. As well, evidence has also shown that cognitive behavioral interventions at schools have been effective in reducing aggression with small effects (*d* = 0.22) [77].

Education can able to improve the performance of clinical staff in reducing the escalation of aggressive behavior [78]. And it even leads to a change in attitude and understanding as well as more confidence in the management of aggression in nurses [79]. It is recommended to use this theory in clinical employees who are exposed to aggression for further research.

Although the current research has several strengths, including a theory-based study and a randomized controlled trial, it has certain limitations. Limitations of this study are as follows: (1) this study was conducted in male students so the results may not be generalizable to female students, and it should be noted that Iran's education policy has considered restrictions for the presence of researchers or teachers of the opposite sex in schools. In addition, the enrollment of female students and other grades in the study required a larger sample size and a larger number of schools, which was not possible due to the time and resources allocated to the master's thesis. (2) It was conducted only in the age group of adolescents. (3) Since the questionnaire was completed by the students themselves, social desirability may have occurred.

The results of this study were in favor of the effectiveness of an educational intervention based TPB on improving the determinants of aggression behavior. Since aggression is a social behavior and a change in the process is time-consuming, therefore it is suggested that training be provided in a long follow-up so that students have the opportunity to practice techniques and skills to change their behavior.

## Figures and Tables

**Figure 1:** CONSORT flow diagram.

**Table 1:** Summary of training sessions based on TPB to prevent and control aggression behaviors.

Lesson	Educational method	Educational content
First session	Lecture	Introduction to the goal of intervention and activities. This session was held with the object of breaking the ice of communication-explaining the intervention.
Second session (knowledge, attitude(	Questions and answers session, lecture	The definition of aggression, the symptoms of aggression and situations that cause anger and aggression, and how to control and prevent aggression. Provide statistics on the prevalence and incidence of aggressive behavior in Iran.
Third session )subjective norms)	Role-play Video lecture	Discussing and examining beliefs individual and social and normative beliefs about aggression behaviors. Also, identifying social factors influencing such as parents and siblings' peer influence, teachers, and pressure. Interpersonal skill training and effective communication was held in the presence of parents or a family member and other school staff.
Fourth session (perceived behavioral control)	Video clips, discussion	Anger management skills by using relaxation techniques through breathing, practicing step-by-step relaxation, coping with negative thoughts, and making changes in the environment were teach. One student who was able to control aggressive was invited to talk about experiences of aggression and effects of aggression and the how to control of aggression.
Fifth session	Brain storming, questions and answers, lecture	Problem-solving, self-control, and decision-making skills were taught, and benefits and barriers to aggression prevention were discussed.

**Table 2:** Comparing demographic variables of participants in intervention and control groups.

Variable		Intervention group *N* (%)	Control group *N* (%)	*p* value^∗^
Fathers' education	Illiterate	4 (8.2)	0	0.156
	Elementary	2 (4.1)	0	
	Secondary	8 (16.3)	11 (22.4)	
	Diploma	10 (20.4)	10 (20.4)	
	Graduate study	25 (51)	28 (57.1)	
Mother's education	Illiterate	4 (8.2)	2 (4.1)	0.296
	Elementary	7 (14.3)	2 (4.1)	
	Secondary	10 (20.4)	8 (16.3)	
	Diploma	13 (26.5)	17 (34.7)	
	Graduate study	15 (30.6)	20 (40.8)	
Father's job	Unemployed	4 (8.2)	5 (10.2)	0.114
	Open market	33 (67.3)	23 (46.9)	
	Staff	12 (24.5)	21 (42.9)	
Mother's job	Employed	7 (14.3)	10 (20.4)	0.16
	Housewife	42 (85.7)	39 (79.6)	

^∗^Chi-square.

**Table 3:** Comparison of mean scores on TPB's constructs within and between experimental and control groups of students, pre- and postintervention.

Construct	Group	Preintervention		Postintervention		*p* value (paired *t*-test)	Effect size^b^ (Cohen's *d*)
		Mean	SD	Mean	SD		
Knowledge	Experimental (*n* = 49)	13.65	4.08	21.40	3.46	<0.001^∗∗^	1.97
	Control (*n* = 49**)**	14.65	4.03	14.18	3.84	0.527	
	*p* value^a^	0.241		<0.00^1∗∗^		—	—
Attitudes	Experimental (*n* = 49)	70.92	11.39	80.18	5.77	<0.001^∗∗^	1.76
	Control (*n* = 49)	68.65	10.93	64.30	12.27	0.032	
	*p* value^∗^	0.422		<0.001^∗∗^		—	—
Subjective norms	Experimental (*n* = 49)	15.83	4.21	15.08	3.72	0.151	0.40
	Control (*n* = 49)	16.45	4.54	16.64	3.91	0.789	
	*p* value^∗^	0.555		0.156		—	—
Behavioral intention	Experimental (*n* = 49)	11.06	4.20	14.59	5.06	<0.001^∗∗^	0.06
	Control (*n* = 49)	15.28	6.96	14.93	5.08	0.757	
	*p* value^∗^	0.291		<0.001^∗∗^		—	—
Perceive behavioral control	Experimental (*n* = 49)	90.22	14.40	106	10.90	<0.001^∗∗^	1.43
	Control (*n* = 49)	82.61	15.12	87.18	15.43	0.173	
	*p* value^∗^	0.012^∗∗∗^		<0.001^∗∗^		—	—

^a^Independent sample *t*-test. ^b^Effect size of Cohen's *d*. ^∗∗^*p* < 0.001 and ^∗∗∗^*p* < 0.05.

**Table 4:** Comparison of mean scores of each type of aggressive behaviors between experimental and control groups of students, pre- and postintervention.

Construct	Time	Experimental group (*n* = 49)	Control group (*n* = 49)	*p* value^∗^	Effect size^b^ (Cohen's *d*)
		Mean (SD)	Mean (SD)		
Verbal	Preintervention	15.48 (3.80)	14.77 (3.36)	0.706	0.41
	Postintervention	16.93 (3.17)	14.51 (2.9)	0≥.0001^∗∗^	
Physical	Preintervention	30.42 (7.64)	26.57 (7.71)	0.810	0.32
	Postintervention	32.53 (5.40)	26.24 (5.12)	0≥.0001^∗∗^	
Hostility	Preintervention	25.97 (6.64)	22.38 (6.14)	1	0.26
	Postintervention	27.57 (5.43)	22.38 (5.21)	0≥.0001^∗∗^	
Anger	Preintervention	22.91 (5.20)	20.28 (4.32)	0.240	0.56
	Postintervention	25.46 (3.89)	21.79 (7.79)	0≥.0001^∗∗^	

^∗^Paired *t*-test. ^∗∗^*p* < 0.001.

## Data Availability

Data used in the analysis as well as all programs used for the analysis may be obtained by contacting the corresponding author on reasonable request.
